RETRACTED

# The Influence of ICAM1 3′UTR Gene Polymorphism on the Occurrence and Metastasis of Primary Liver Cancer

**DOI:** 10.1155/2021/7377299

**Published:** 2021-11-26

**Authors:** Li He, Suwen Wang, Xusheng Ma

**Affiliations:** ^1^Houbo College of Xinjiang Medical University, No. 12 of Shengli Road, Karamay, Xinjiang, China; ^2^Shihezi University School of Medicine, Beier Road, Shihezi, Xinjiang, China

## Abstract

**Objective:**

In this study, we explored the influence of single nucleotide polymorphism (SNP) in the noncoding region of intercellular adhesion molecule 1 (ICAM1) gene on the occurrence and metastasis of primary hepatocellular carcinoma (PHC).

**Methods:**

Sanger sequencing was used to analyze the genotypes of rs3093032, rs923366, and rs281437 locus in the 3′untranslated region (UTR) of the *ICAM1* gene. The level of plasma ICAM1 was analyzed by enzyme-linked immunosorbent assay (ELISA).

**Results:**

After adjusting for risk factors such as BMI, smoking, drinking, family history of tumors, and hepatitis B virus test results, the CT genotype at rs3093032 of the *ICAM1* gene (OR = 0.19, 95% CI: 0.08-0.44, *P* < 0.01), dominance model (OR = 0.23, 95% CI: 0.11-0.48, *P* < 0.01), and T allele (OR = 0.27, 95% CI: 0.14-0.53, *P* < 0.01) were related to the reduced risk of PHC susceptibility. rs923366 locus CT genotype (OR = 0.63, 95% CI: 0.44-0.90, *P* = 0.01), TT genotype (OR = 0.23, 95% CI: 0.10-0.53, *P* < 0.01), dominant model (OR = 0.55, 95% CI: 0.39-0.77, *P* < 0.01), recessive model (OR = 0.28, 95% CI: 0.12-0.62, *P* < 0.01), and T allele (OR = 0.55, 95% CI: 0.42-0.73, *P* < 0.01) were related to a reduction in the risk of PHC susceptibility. rs281437 locus CT genotype (OR = 2.08, 95% CI: 1.40-3.09, *P* < 0.01), TT genotype (OR = 5.20, 95% CI: 2.22-12.17, *P* < 0.01), dominant model (OR = 2.45, 95% CI: 1.69-3.54, *P* < 0.01), recessive model (OR = 4.32, 95% CI: 1.86-10.06, *P* < 0.01), and T allele (OR = 2.46, 95% CI: 1.79-3.38, *P* < 0.01) were significantly related to the increased risk of PHC susceptibility. SNPs at rs3093032, rs923366, and rs281437 of the *ICAM1* gene were significantly correlated with TNM stage and tumor metastasis of PHC patients (*P* < 0.05).

**Conclusion:**

SNPs at rs3093032, rs923366, and rs281437 in the 3′UTR region of the *ICAM1* gene are related to the occurrence and metastasis of PHC.

## 1. Introduction

Primary hepatocellular carcinoma (PHC) is one of the most common malignant tumors in the world, and its morbidity and mortality are among the top malignant tumors in the world [1, 2]. The treatment of PHC mainly includes radical surgery, hepatic artery embolization chemotherapy, radiotherapy, and local radiofrequency ablation, but it is easy to relapse after treatment and the prognosis is poor [3–5].

RETRACTED

The cause and pathogenesis of hepatocellular carcinoma have not yet been fully elucidated. With the progress of molecular biology, virology, and genetics, researchers have found that the occurrence of hepatocellular carcinoma is related to the interaction of environmental and genetic factors [6, 7]. Important risk factors for hepatocellular carcinoma include chronic hepatitis B virus and chronic hepatitis C virus infection, alcohol abuse, chromosomal instability, oxidative damage, DNA methylation genetic signal transduction pathway obstacles, and gene polymorphisms. Therefore, to study the molecular pathological mechanism of PHC and to find new treatment methods at the gene level are of great significance for the prevention and treatment of PHC.

Intercellular adhesion molecule 1 (ICAM1) is a transmembrane single-chain glycoprotein with a molecular weight of 90-115 kD. It belongs to the immunoglobulin superfamily. It has five immunoglobulin structures and a transmembrane structure. It is expressed in leukocytes, fibroblasts, epithelial cells, and other cells [8, 9]. The *ICAM1* gene is located on the human chromosome 19p13.2, which consists of 7 exons, 6 introns, 2.4 kb upstream sequence, and 1.5 kb 3′ noncoding RNA sequence. The rs3093032 site is located at 10285660 bp, the rs923366 site is located at 10286547 bp, and the rs281437 site is located at 10286562 bp, all located in the 3′UTR region of the *ICAM1* gene.

In this study, rs3093032 locus, rs923366 locus, and rs281437 locus were selected for research to explore their correlation with the occurrence and metastasis of PHC and provide clinical value for the prevention and treatment of PHC.

## 2. Methods

### 2.1. Ethics Statement

This study followed the “Declaration of Helsinki” and was carried out with the approval of the ethics committee. The subjects signed a written informed consent.

### 2.2. Subjects

A collection of 290 PHC patients who were clinically admitted in the National Human Genetic Resources Sharing Service Platform from 2013 to 2016 were used as the research objects. All patients included in the study were diagnosed as PHC through clinical, imaging, and pathology. Among them, there were 163 male PHC patients and 127 female patients. Inclusion criteria are as follows: (1) the diagnostic criteria of PHC conformed to practice guidelines for the pathological diagnosis of primary liver cancer [10]; (2) no adjuvant treatment was performed before surgery. Exclusion criteria are as follows: (1) patients who had received radiotherapy and chemotherapy; (2) patients with a history of blood transfusion; (3) patients with other vital organ diseases such as heart, lung, and kidney; (4) patients with hyperlipidemia; (5) patients with hypertension; and (6) patients with diabetes. Two hundred and ninety non-PHC patients with no history of blood transfusion, no heart, lung, or kidney disease, no hyperlipidemia, and no hypertension or diabetes were recruited as the control group, including 166 males and 124 females. A questionnaire was designed to collect the basic information of the subjects; the content of the questionnaire included the patient's age, gender, body mass index (BMI), smoking, drinking, tumor family history, hepatitis B virus, and other information.

RETRACTED

### 2.3. Selection of SNP Sites

According to the variation tool in the National Center for Biotechnology Information (NCBI) database, the minor allele frequency (MAF) > 0.05 in the 3′UTR region of the *ICAM1* gene was selected for research.

### 2.4. Genotype Analysis of SNP Locus of the *ICAM1* Gene

We collected 5 mL of peripheral venous blood from each subject, and genomic DNA was extracted from peripheral blood leukocytes using TIANamp Blood DNA Kit (Tiangen Biotech, Beijing, China). According to the sequence information of 100 bp upstream and downstream of the SNP site in the database of dbSNP (https://www.ncbi.nlm.nih.gov/snp/), primer sequences were designed using Primer-BLAST. The rs3093032 site primer sequence was 5′-ACA TAG CCC CAC CAT GAG GA-3′ (forward) and 5′-ACA TGT CTA TGG AGG GCC AC-3′ (reverse). The rs923366 site primer sequence was 5′-CAG CTT TGG AAG CCT CAT CCG-3′ (forward) and 5′-GTG ACA CCT CCC CTC AAC TC-3′ (reverse). The rs281437 site primer sequence was 5′-GCC TCA GCC TTG TGT GAG TTG-3′ (forward) and 5′-GAT CAG GCT GTG GCT GCT TAG-3′ (reverse). The primers were synthesized by Shanghai Sijia Biotechnology Co., Ltd. (Shanghai, China), and then, PCR reaction was performed. The PCR reaction system consists of 2.5 *μ*L 10x buffer, 0.5 *μ*L dNTP (10 mmol/L), 5 *μ*L each of forward primer and reverse primer, 5 *μ*L DNA template, 2 U Taq enzyme, and ddH_2_O to keep the total volume at 25 *μ*L. The PCR reaction conditions were 94°C predenaturation for 2 minutes and then 94°C, 30 s, 60°C, 35 s, 72°C, 45 s, and repeated 30 cycles. After the PCR amplification was completed, the products were sequenced by Shanghai Sijia Biotechnology Co., Ltd. (Shanghai, China) and compared with the dbSNP database based on the sequencing results, and the subject's genotype was determined based on the comparison results.

### 2.5. Enzyme-Linked Immunosorbent Test (ELISA)

The ICAM1 (soluble) Human ELISA Kit (Thermo Fisher Scientific, Waltham, USA) was used to detect the plasma ICAM1 level of the subjects. Using the detected OD_450_ as the ordinate and the concentration of the standard as the abscissa, we drew a standard curve and calculated the concentration of soluble ICAM1 in the plasma sample according to the OD_450_ value, and each sample was tested 3 times.

RETRACTED

### 2.6. Statistical Analysis

The *χ*^2^ test was used to evaluate the differences between groups of categorical variables [*n* (%)], and the *t-*test and one-way ANOVA were used to evaluate the differences between groups of continuous variables (mean ± SD). Whether the genotype frequency accords with Hardy-Weinberg equilibrium was evaluated by the *χ*^2^ test. Logistic regression was used to analyze the correlation between SNPs at rs3093032, rs923366, and rs281437 in the *ICAM1* gene and PHC susceptibility, the odds ratio (OR) and 95% confidence interval (CI) were calculated, and the risk factors of PHC in the single factor logistic regression analysis were adjusted. SPSS 26.0 (SPSS, Chicago, IL, USA) was used for statistical analysis. All statistical tests were two-sided tests. *P* < 0.05 indicated that the difference was statistically significant.

## 3. Results

### 3.1. Clinical Characteristics of Patients with Primary Liver Cancer and the Control Group

The clinical characteristics of 290 PHC patients and the control group are compared in Table 1. The results of one-way ANOVA showed that body mass index (BMI), smoking, drinking, family history of tumors, and hepatitis B virus test results were related to PHC susceptibility, including BMI ≥ 25 kg/m^2^, smoking, drinking, family history of tumors, and hepatitis B virus positive which were risk factors for PHC (*P* < 0.05) (Table 1).

### 3.2. *ICAM1* Gene Polymorphism Was Associated with PHC Susceptibility

First, we analyzed the genotype frequencies of *ICAM1* gene rs3093032, rs923366, and rs281437 locus in the control group. The results showed that the control group *ICAM1* gene rs3093032, rs923366, and rs281437 locus genotype frequencies were in accordance with the Hardy-Weinberg equilibrium (*P* = 0.11, *P* = 0.23, and *P* = 0.07) (data not listed in Table 2). According to ICAM1 gene rs3093032 locus, rs923366 locus, and rs281437 locus allele frequency, the minimum sample size of the PHC and control groups was 63 cases/63 cases, 108 cases/108 cases, and 89 cases/89 cases, respectively.

The analysis results showed that taking the CC genotype at rs3093032 as a reference, after adjusting for risk factors such as BMI, smoking, drinking, family history of tumors, and hepatitis B virus test results, the CT genotype (OR = 0.19, 95% CI: 0.08-0.44, *P* < 0.01) and the dominant model (OR = 0.23, 95% CI: 0.11-0.48, *P* < 0.01) were related to the reduced risk of PHC susceptibility, and the PHC susceptibility risk of T allele carriers was 0.27 times than that of C allele carriers (95% CI: 0.14-0.53, *P* < 0.01).

RETRACTED

Taking the CC allele at rs923366 as a reference, after adjusting for risk factors such as BMI, smoking, drinking, family history of tumors, and hepatitis B virus test results, the CT genotype (OR = 0.63, 95% CI: 0.44-0.90, *P* = 0.01), TT genotype (OR = 0.23, 95% CI: 0.10-0.53, *P* < 0.01), dominant model (OR = 0.55, 95% CI: 0.39-0.77, *P* < 0.01), recessive model (OR = 0.28, 95% CI: 0.12-0.62, *P* < 0.01), and the risk of PHC susceptibility was reduced. The PHC susceptibility risk of T allele carriers was 0.55 times than that of C allele carriers (95% CI: 0.42-0.73, *P* < 0.01).

Compared with the CC genotype at rs281437, CT genotype (OR = 2.08, 95% CI: 1.40-3.09, *P* < 0.01), TT genotype (OR = 5.20, 95% CI: 2.22-12.17, *P* < 0.01), the dominant model (OR = 2.45, 95% CI: 1.69-3.54, *P* < 0.01), and the recessive model (OR = 4.32, 95% CI: 1.86-10.06, *P* < 0.01) were associated with increased risk of PHC susceptibility, and the PHC susceptibility risk of T allele carriers was 2.46 times than that of the C allele (95% CI: 1.79-3.38, *P* < 0.01) (Table 2).

### 3.3. Stratified Analysis

In order to further refine the relationship between genetic factors and PHC susceptibility in different populations, we conducted a stratified analysis for the population's age, gender, body mass index (BMI), smoking, drinking, family history of tumors, and hepatitis B virus test results. The analysis results showed that only young people (age < 60 years), elderly people (age ≥ 60 years), male, BMI < 25 kg/m^2^, BMI ≥ 25 kg/m^2^, smokers, nonsmokers, drinkers, nondrinkers, no family history of cancer, and carriers of CT+TT genotype at rs3093032 had a lower risk of susceptibility to PHC than CC genotype (*P* < 0.05) (Table 3).

Young people (age < 60 years), elderly people (age ≥ 60 years), female, BMI < 25 kg/m^2^, BMI ≥ 25 kg/m^2^, nonsmokers, drinkers, nondrinkers, no family history of cancer, hepatitis B virus-positive people, and carriers of CT+TT genotype at rs923366 had a lower risk of susceptibility to PHC than CC genotype (*P* < 0.05) (Table 4).

Young people, elderly people, female, BMI < 25 kg/m^2^, BMI ≥ 25 kg/m^2^, smokers, nonsmokers, drinkers, nondrinkers, no family history of cancer, hepatitis B virus-positive people, hepatitis B virus-negative people, and carriers of rs281437 CT+TT genotype had higher risk of susceptibility to PHC than CC genotype (*P* < 0.05) (Table 5).

### 3.4. Correlation between *ICAM1* Gene Polymorphism and TNM Stage

SNPs at rs3093032, rs923366, and rs281437 of the *ICAM1* gene were significantly correlated with TNM stage (*P* < 0.05) (Table 6). The progress of PHC patients with CT+TT genotype and CC genotype at rs3093032 was low, the progress of PHC patients with CT+TT genotype and CC genotype at rs923366 was low, and PHC patients with CT+TT genotype and CC genotype at rs281437 had a high degree of progression. This showed that the SNPs at rs3093032, rs923366, and rs281437 of the *ICAM1* gene were associated with tumor progression in PHC patients.

RETRACTED

### 3.5. The Correlation between *ICAM1* Gene Polymorphism and Tumor Metastasis

*ICAM1* gene rs3093032 locus and rs923366 locus CT+TT genotype had lower risk of tumor metastasis than CC genotype PHC patients (*P* < 0.05). The risk of tumor metastasis in patients with CT+TT genotype PHC at rs281437 was significantly higher than that of patients with CC genotype PHC (*P* < 0.05) (Table 7).

### 3.6. Plasma ICAM1 Levels in PHC Patients Were Abnormally Elevated, and *ICAM1* Gene Polymorphisms Were Related to Plasma ICAM1 Levels

The plasma ICAM1 level of subjects was detected by ELISA, and the results showed that the plasma ICAM1 level of PHC patients was abnormally increased (*P* < 0.01, Figure 1(a)). We observed that the differences in plasma ICAM1 levels of *ICAM1* gene rs3093032, rs923366, and rs281437 in plasma of PHC patients and the control group were statistically significant (*P* < 0.05). The plasma ICAM1 level of subjects with CT+TT genotype at rs3093032 was significantly lower than that of subjects with CC genotype (*P* < 0.01, Figure 1(b)). The plasma ICAM1 level of subjects with CT+TT genotype at rs923366 locus was significantly lower than that of subjects with CC genotype (*P* < 0.01, Figure 1(c)). The plasma ICAM1 level of subjects with CT+TT genotype at rs281437 locus was significantly higher than that of subjects with CC genotype (*P* < 0.05, Figure 1(d)).

### 3.7. Correlation between Plasma ICAM1 Level and Tumor Progression and Metastasis in PHC Patients

We further analyzed the correlation between plasma ICAM1 level in PHC patients and tumor progression and metastasis, and the results showed that plasma ICAM1 levels in PHC patients with tumor progression were higher (*P* < 0.01, Figure 2(a)). Compared with PHC patients without tumor metastasis, we detected higher levels of ICAM1 in the plasma of patients with tumor metastasis (*P* < 0.01, Figure 2(b)).

## 4. Discussion

At present, surgical resection was still the most effective treatment for liver cancer, but due to the multifocality of liver cancer, vascular invasion, combined with liver cirrhosis, a small number of patients were suitable for surgical treatment [11, 12]. With the improvement of surgery, chemotherapy, and radiotherapy, the survival rate of liver cancer patients had been greatly improved, but distant metastasis was the most important factor affecting their prognosis [13]. Therefore, research on the pathogenesis of liver cancer and a correct understanding of the mechanism and mode of liver cancer metastasis were essential for formulating a reasonable treatment plan and adopting targeted intervention measures to improve survival.

RETRACTED

ICAM1 belongs to the immunoglobulin superfamily. It is a single-transmembrane single-chain glycoprotein. There are 5 immunoglobulin structural regions in the extracellular region, of which the I region binds to LFA-1 and the III region and complement receptor-3 (CR3 or Mac-1), and ICAM1 works by combining with LFA-1 and Mac-1 [14–16]. ICAM1 is widely present in white blood cells, monocytes, peripheral blood lymphocytes, vascular endothelial cells, etc. [17]. Studies had found that ICAM1 could bind to LFA-1 and Mac-1 to inhibit the activation and transmission of the second signal system of CTL and NK and made cytotoxic T cells, natural killer cells, and macrophages lost their ability to kill tumor cells, which escaped the body's cellular immune surveillance [14, 18, 19].

In this study, we found that the plasma ICAM1 level of PHC patients was significantly higher than that of the control group, and the plasma ICAM1 level of PHC patients with tumor progression and metastasis was higher, which was consistent with the results of Zhu et al. [20]. The researcher found that ICAM1 may be a potential serum biomarker for liver cancer diagnosis in 236 patients with hepatocellular carcinoma (HCC) undergoing hepatectomy. It was also an independent predictor of DFS and OS after surgical resection and is expected to provide important reference value for the prediction of intrahepatic and extrahepatic metastasis. In addition, Guo et al. [21] found that the increase of ICAM1 expression level was related to the development of HCC complication portal vein tumor thrombosis (PVTT) and poor prognosis. It reminded us that ICAM1 played an important role in the occurrence and development of PHC.

We knew that the occurrence and development of PHC were closely related to genetic factors and environmental factors. At present, there was little research on ICAM1 gene polymorphism and the occurrence and development of PHC. Chen et al. [22] studied 305 HCC patients and 613 controls and found that the interaction between *ICAM1* gene rs5498 site SNP and the environment was related to the susceptibility of liver cancer, which could be used as a marker of the risk of vascular invasion in smokers with liver cancer. In this study, we found that SNPs at rs3093032, rs923366, and rs281437 in the 3′UTR region of the *ICAM1* gene were significantly related to the risk of PHC susceptibility, tumor progression, and metastasis. Combined with the bioinformatics prediction, we speculated that the rs3093032 locus was located at the predicted junction of hsa-miR-4648 and the 3′UTR of the *ICAM1* gene, the rs923366 site was located at the predicted binding site of hsa-miR-1299 and hsa-miR-875-3p with the 3′UTR of the *ICAM1* gene, and the rs281437 site was located at the predicted binding site of hsa-miR-3667-5p, hsa-miR-4684-3p, and hsa-miR-4696 and *ICAM1* gene 3′UTR. Whether these SNPs affected the expression of ICAM1 and the role of microRNAs in it needed further study.

RETRACTED

In conclusion, SNPs at rs3093032, rs923366, and rs281437 in the 3′UTR region of the *ICAM1* gene are related to the occurrence and metastasis of PHC and may be new targets for PHC prevention and treatment.

## Figures and Tables

**Figure 1:** Results of plasma ICAM1 level detection: (a) plasma ICAM1 level of PHC patients compared with control subjects; (b) comparison of plasma ICAM1 levels between subjects with CT+TT genotype at rs3093032 and subjects with CC genotype; (c) comparison of plasma ICAM1 levels in subjects with CT+TT genotype at rs923366 locus and subjects with CC genotype; (d) comparison of plasma ICAM1 levels in subjects with CT+TT genotype at rs281437 locus and subjects with CC genotype.

**Figure 2:** The correlation between plasma ICAM1 level and tumor progression and metastasis in PHC patients: (a) comparison of plasma ICAM1 levels in PHC patients with different TNM stages; (b) comparison of plasma ICAM1 levels between PHC patients with tumor metastasis and without tumor metastasis.

**Table 1:** Comparison of clinical characteristics between PHC patients and controls.

Characteristics	PHC (*n* = 290)	Control (*n* = 290)	OR (95% CI)	*P* value
Age [*n* (%)]				
<60	136 (46.90%)	140 (48.28%)	1.00 (reference)	
≥60	154 (53.10%)	150 (51.72%)	1.06 (0.76-1.46)	0.80
Gender [*n* (%)]				
Male	163 (56.21%)	166 (57.24%)	1.00 (reference)	
Female	127 (43.79%)	124 (42.76%)	1.04 (0.75-1.45)	0.87
BMI [kg/m^2^, *n* (%)]				
<25	147 (50.69%)	175 (60.34%)	1.00 (reference)	
≥25	143 (49.31%)	115 (39.66%)	1.48 (1.07-2.06)	0.02
Smoking [*n* (%)]				
No	125 (43.10%)	174 (60.00%)	1.00 (reference)	
Yes	165 (56.90%)	116 (40.00%)	1.98 (1.42-2.76)	<0.01
Drinking [*n* (%)]				
No	118 (40.69%)	156 (53.79%)	1.00 (reference)	
Yes	172 (59.31%)	134 (46.21%)	1.70 (1.22-2.36)	<0.01
Family history of tumors [*n* (%)]				
No	236 (81.38%)	278 (95.86%)	1.00 (reference)	
Yes	54 (18.62%)	12 (4.14%)	5.30 (2.77-10.15)	<0.01
Hepatitis B virus [*n* (%)]				
Positive	53 (18.28%)	255 (87.93%)	1.00 (reference)	
Negative	237 (81.72%)	35 (12.07%)	5.06 (4.12-6.17)	<0.01
TNM staging [*n* (%)]				
I	42 (14.48%)			
II	75 (25.86%)			
III	86 (29.66%)			
IV	87 (30.00%)			
Metastasis				
Yes	168 (57.93%)			
No	122 (42.07%)			

PHC: primary hepatocellular carcinoma; OR: odds ratio; CI: confidence interval; BMI: body mass index; TNM: tumor-node-metastasis.

RETRACTED

**Table 2:** *ICAM1* gene rs3093032 locus, rs923366 locus, rs281437 locus genotype, genetic model, allele frequency, and PHC susceptibility.

	PHC (*n* = 290)	Control (*n* = 290)	OR (95% CI)^∗^	*P* value
rs3093032				
CC	281 (96.90%)	254 (87.59%)	1.00 (reference)	
CT	7 (2.41%)	33 (11.38%)	0.19 (0.08-0.44)	<0.01
TT	2 (0.69%)	3 (1.03%)	0.60 (0.10-3.64)	0.91
CT+TT	9 (3.10%)	36 (12.41%)	0.23 (0.11-0.48)	<0.01
CC+CT	288 (99.31%)	287 (98.97%)	1.00 (reference)	
TT	2 (0.69%)	3 (1.03%)	0.66 (0.11-4.01)	0.65
C	569 (98.10%)	541 (93.28%)	1.00 (reference)	
T	11 (1.90%)	39 (6.72%)	0.27 (0.14-0.53)	<0.01
rs923366				
CC	195 (67.24%)	154 (53.10%)	1.00 (reference)	
CT	87 (30.00%)	109 (37.59%)	0.63 (0.44-0.90)	0.01
TT	8 (2.76%)	27 (9.31%)	0.23 (0.10-0.53)	<0.01
CT+TT	95 (32.76%)	136 (46.90%)	0.55 (0.39-0.77)	<0.01
CC+CT	282 (97.24%)	263 (90.69%)	1.00 (reference)	
TT	8 (2.76%)	27 (9.31%)	0.28 (0.12-0.62)	<0.01
C	477 (82.24%)	417 (71.90%)	1.00 (reference)	
T	103 (17.76%)	163 (28.10%)	0.55 (0.42-0.73)	<0.01
rs281437				
CC	177 (61.03%)	230 (79.31%)	1.00 (reference)	
CT	85 (29.31%)	53 (18.28%)	2.08 (1.40-3.09)	<0.01
TT	28 (9.66%)	7 (2.41%)	5.20 (2.22-12.17)	<0.01
CT+TT	113 (38.97%)	60 (20.69%)	2.45 (1.69-3.54)	<0.01
CC+CT	262 (90.34%)	283 (97.59%)	1.00 (reference)	
TT	28 (9.66%)	7 (2.41%)	4.32 (1.86-10.06)	<0.01
C	439 (75.69%)	513 (88.45%)	1.00 (reference)	
T	141 (24.31%)	67 (11.55%)	2.46 (1.79-3.38)	<0.01

^∗^Adjust factors such as BMI, smoking, drinking, family history of tumors, and hepatitis B virus. OR: odds ratio; CI: confidence interval.

**Table 3:** Stratified analysis of the correlation between SNP at rs3093032 of the *ICAM1* gene and PHC susceptibility risk.

	PHC (*n* = 290)	Control (*n* = 290)	OR (95% CI)^∗^	*P* value
Age [years, *n* (%)]				
<60				
CC	133 (97.79%)	122 (87.14%)	1.00 (reference)	
CT+TT	3 (2.21%)	18 (12.86%)	0.15 (0.04-0.53)	<0.01
≥60				
CC	148 (96.10%)	132 (88.00%)	1.00 (reference)	
CT+TT	6 (3.90%)	18 (12.00%)	0.30 (0.12-0.77)	0.02
Gender [*n* (%)]				
Male				
CC	157 (96.32%)	139 (83.73%)	1.00 (reference)	
CT+TT	6 (3.68%)	27 (16.27%)	0.20 (0.08-0.49)	<0.01
Female				
CC	124 (97.64%)	115 (92.74%)	1.00 (reference)	
CT+TT	3 (2.36%)	9 (7.26%)	0.31 (0.08-1.17)	0.13
BMI [kg/m^2^, *n* (%)]				
<25				
CC	144 (97.96%)	153 (87.43%)	1.00 (reference)	
CT+TT	3 (2.04%)	22 (12.57%)	0.15 (0.04-0.49)	<0.01
≥25				
CC	137 (95.80%)	101 (87.83%)	1.00 (reference)	
CT+TT	6 (4.20%)	14 (12.17%)	0.32 (0.12-0.85)	0.03
Smoking [*n* (%)]				
No				
CC	123 (98.40%)	151 (86.78%)	1.00 (reference)	
CT+TT	2 (1.60%)	23 (13.22%)	0.11 (0.03-0.46)	<0.01
Yes				
CC	158 (95.76%)	103 (88.79%)	1.00 (reference)	
CT+TT	7 (4.24%)	13 (11.21%)	0.35 (0.14-0.91)	0.04
Drinking [*n* (%)]				
No				
CC	118 (99.16%)	139 (89.10%)	1.00 (reference)	
CT+TT	1 (0.84%)	17 (10.90%)	0.07 (0.01-0.53)	<0.01
Yes				
CC	163 (95.32%)	115 (85.82%)	1.00 (reference)	
CT+TT	8 (4.68%)	19 (14.18%)	0.30 (0.13-0.70)	<0.01
Family history of cancer [*n* (%)]				
No				
CC	229 (97.45%)	243 (87.41%)	1.00 (reference)	
CT+TT	6 (2.55%)	35 (%)	0.18 (0.08-0.44)	<0.01
Yes				
CC	52 (94.55%)	11 (91.67%)	1.00 (reference)	
CT+TT	3 (5.45%)	1 (8.33%)	0.64 (0.06-6.69)	0.70
Hepatitis B virus [*n* (%)]				
Negative				
CC	51 (96.23%)	222 (87.06%)	1.00 (reference)	
CT+TT	2 (3.77%)	33 (12.94%)	0.26 (0.06-1.14)	0.09
Positive				
CC	230 (97.05%)	32 (91.43%)	1.00 (reference)	
CT+TT	7 (2.95%)	3 (8.57%)	0.33 (0.08-1.32)	0.24

^∗^Adjust factors such as BMI, smoking, drinking, family history of tumors, and hepatitis B virus. OR: odds ratio; CI: confidence interval.

RETRACTED

**Table 4:** Stratified analysis of the correlation between SNP at rs923366 of the *ICAM1* gene and PHC susceptibility risk.

	PHC (*n* = 290)	Control (*n* = 290)	OR (95% CI)^∗^	*P* value
Age [years, *n* (%)]				
<60				
CC	90 (66.18%)	75 (53.57%)	1.00 (reference)	
CT+TT	46 (33.82%)	65 (46.43%)	0.59 (0.36-0.96)	0.04
≥60				
CC	105 (68.18%)	79 (52.67%)	1.00 (reference)	
CT+TT	49 (31.82%)	71 (47.33%)	0.52 (0.33-0.83)	<0.01
Gender [*n* (%)]				
Male				
CC	99 (60.74%)	96 (57.83%)	1.00 (reference)	
CT+TT	64 (39.26%)	70 (42.17%)	0.89 (0.57-1.38)	0.67
Female				
CC	96 (75.59%)	58 (46.77%)	1.00 (reference)	
CT+TT	31 (24.41%)	66 (53.23%)	0.28 (0.17-0.49)	<0.01
BMI [kg/m^2^, *n* (%)]				
<25				
CC	108 (73.47%)	92 (52.57%)	1.00 (reference)	
CT+TT	39 (26.53%)	83 (47.43%)	0.40 (0.25-0.64)	<0.01
≥25				
CC	87 (60.84%)	62 (53.91%)	1.00 (reference)	
CT+TT	56 (39.16%)	53 (46.09%)	0.75 (0.46-1.24)	0.32
Smoking [*n* (%)]				
No				
CC	93 (74.40%)	93 (53.45%)	1.00 (reference)	
CT+TT	32 (25.60%)	81 (46.55%)	0.40 (0.24-0.65)	<0.01
Yes				
CC	102 (61.82%)	61 (52.59%)	1.00 (reference)	
CT+TT	63 (38.18%)	55 (47.41%)	0.69 (0.42-1.11)	0.16
Drinking [*n* (%)]				
No				
CC	83 (69.75%)	90 (57.69%)	1.00 (reference)	
CT+TT	36 (30.18%)	66 (42.31%)	0.59 (0.36-0.98)	0.04
Yes				
CC	112 (65.50%)	64 (47.76%)	1.00 (reference)	
CT+TT	59 (34.50%)	70 (52.24%)	0.48 (0.30-0.77)	<0.01
Family history of cancer [*n* (%)]				
No				
CC	158 (67.23%)	146 (52.52%)	1.00 (reference)	
CT+TT	77 (32.77%)	132 (47.48%)	0.54 (0.38-0.77)	<0.01
Yes				
CC	37 (67.27%)	8 (66.67%)	1.00 (reference)	
CT+TT	18 (32.77%)	4 (33.33%)	0.97 (0.26-3.66)	0.97
Hepatitis B virus [*n* (%)]				
Negative				
CC	36 (67.92%)	139 (54.51%)	1.00 (reference)	
CT+TT	17 (32.08%)	116 (45.49%)	0.57 (0.30-1.06)	0.10
Positive				
CC	159 (67.09%)	15 (42.86%)	1.00 (reference)	
CT+TT	78 (32.91%)	20 (57.14%)	0.37 (0.18-0.76)	<0.01

^∗^Adjust factors such as BMI, smoking, drinking, family history of tumors, and hepatitis B virus. OR: odds ratio; CI: confidence interval.

RETRACTED

**Table 5:** Stratified analysis of the correlation between SNP at rs281437 locus of the *ICAM1* gene and PHC susceptibility risk.

	PHC (*n* = 290)	Control (*n* = 290)	OR (95% CI)^∗^	*P* value
Age [years, *n* (%)]				
<60				
CC	82 (60.29%)	114 (81.43%)	1.00 (reference)	
CT+TT	54 (39.71%)	26 (18.57%)	2.89 (1.67-4.99)	<0.01
≥60				
CC	95 (61.69%)	116 (77.33%)	1.00 (reference)	
CT+TT	59 (38.31%)	34 (22.67%)	2.12 (1.28-3.50)	<0.01
Gender [*n* (%)]				
Male				
CC	111 (68.10%)	127 (76.51%)	1.00 (reference)	
CT+TT	52 (31.90%)	39 (23.49%)	1.53 (0.94-2.48)	0.11
Female				
CC	66 (1.97%)	103 (83.06%)	1.00 (reference)	
CT+TT	61 (48.03%)	21 (16.94%)	4.53 (2.53-8.13)	<0.01
BMI [kg/m^2^, *n* (%)]				
<25				
CC	85 (57.82%)	136 (77.71%)	1.00 (reference)	
CT+TT	62 (42.18%)	39 (22.29%)	2.54 (1.57-4.13)	<0.01
≥25				
CC	92 (64.34%)	94 (81.74%)	1.00 (reference)	
CT+TT	51 (35.66%)	21 (18.26%)	2.48 (1.38-4.45)	<0.01
Smoking [*n* (%)]				
No				
CC	72 (57.60%)	129 (71.14%)	1.00 (reference)	
CT+TT	53 (42.40%)	45 (25.86%)	2.11 (1.29-3.45)	<0.01
Yes				
CC	105 (63.64%)	101 (87.07%)	1.00 (reference)	
CT+TT	60 (36.36%)	15 (12.93%)	3.85 (2.05-7.21)	<0.01
Drinking [*n* (%)]				
No				
CC	79 (66.39%)	127 (81.41%)	1.00 (reference)	
CT+TT	40 (33.61%)	29 (18.59%)	2.22 (1.27-3.86)	<0.01
Yes				
CC	98 (57.31%)	103 (76.87%)	1.00 (reference)	
CT+TT	73 (42.69%)	31 (23.13%)	2.48 (1.50-4.09)	<0.01
Family history of cancer [*n* (%)]				
No				
CC	141 (60.00%)	220 (79.14%)	1.00 (reference)	
CT+TT	94 (40.00%)	58 (20.86%)	2.53 (1.71-3.73)	<0.01
Yes				
CC	36 (65.45%)	10 (83.33%)	1.00 (reference)	
CT+TT	19 (34.55%)	2 (16.67%)	2.64 (0.52-13.29)	0.39
Hepatitis B virus [*n* (%)]				
Negative				
CC	31 (58.49%)	202 (79.22%)	1.00 (reference)	
CT+TT	22 (41.51%)	53 (20.78%)	2.71 (1.45-5.05)	<0.01
Positive				
CC	146 (61.60%)	28 (80.00%)	1.00 (reference)	
CT+TT	91 (38.40%)	7 (20.00%)	2.49 (1.05-5.94)	0.03

^∗^Adjust factors such as BMI, smoking, drinking, family history of tumors, and hepatitis B virus. OR: odds ratio; CI: confidence interval.

**Table 6:** The correlation between the different genotypes at rs3093032, rs923366, and rs281437 of the *ICAM1* gene and TNM stage.

	III/IV (*n* = 173)	I/II (*n* = 117)	OR (95% CI)^∗^	*P* value
rs3093032				
CC	171 (98.84%)	110 (94.02%)	1.00 (reference)	
CT+TT	2 (1.16%)	7 (5.98%)	0.18 (0.04-0.90)	0.04
rs923366				
CC	130 (75.14%)	65 (55.56%)	1.00 (reference)	
CT+TT	43 (24.86%)	52 (44.44%)	0.41 (0.25-0.68)	<0.01
rs281437				
CC	78 (45.09%)	99 (84.62%)	1.00 (reference)	
CT+TT	95 (54.91%)	18 (15.38%)	6.70 (3.73-12.02)	<0.01

^∗^Adjust factors such as BMI, smoking, drinking, family history of tumors, and hepatitis B virus. OR: odds ratio; CI: confidence interval.

RETRACTED

**Table 7:** Correlation between different genotypes at rs3093032, rs923366, and rs281437 of the *ICAM1* gene and metastasis.

	Metastasis (*n* = 168)	Nonmetastasis (*n* = 122)	OR (95% CI)^∗^	*P* value
rs3093032				
CC	166 (98.81%)	115 (94.26%)	1.00 (reference)	
CT+TT	2 (1.19%)	7 (5.74%)	0.20 (0.04-0.97)	0.03
rs923366				
CC	126 (75.00%)	69 (56.56%)	1.00 (reference)	
CT+TT	42 (25.00%)	53 (43.44%)	0.43 (0.26-0.72)	<0.01
rs281437				
CC	74 (44.05%)	103 (84.43%)	1.00 (reference)	
CT+TT	94 (55.95%)	19 (15.57%)	6.89 (3.87-12.26)	<0.01

^∗^Adjust factors such as BMI, smoking, drinking, family history of tumors, and hepatitis B virus. OR: odds ratio; CI: confidence interval.

## Data Availability

The data used during the present study are available from the corresponding author upon reasonable request.
